# Relationship of the high proportion of suicidal acts involving ingestion of pesticides to the low male-to-female ratio of suicide rates in China

**DOI:** 10.1017/S2045796020000244

**Published:** 2020-04-07

**Authors:** Yongsheng Tong, Michael R. Phillips, Yi Yin, Zhichao Lan

**Affiliations:** 1 Beijing Suicide Research and Prevention Center, Beijing Hui Long Guan Hospital, Beijing, China; 2 WHO Collaborating Center for Research and Training in Suicide Prevention, Beijing, China; 3 Peking University HuiLongGuan Clinical Medical School, Beijing, China; 4 Shanghai Mental Health Center, Shanghai Jiao Tong University School of Medicine, Shanghai, China; 5 Departments of Psychiatry and Epidemiology, Columbia University, New York, United States; 6 Center of Disease Control and Prevention of Meixian County, Shananxi Province, China

**Keywords:** Case-fatality, China, gender ratio, pesticide, suicide rates

## Abstract

**Aims:**

The 2014 World Health Organization report on global suicide identified large differences in the male-to-female ratio of suicide rates between countries: most high-income countries (HICs) report ratios of 3:1 or higher while many low- and middle-income countries (LMICs) – including China and India – report ratios of less than 1.5:1. Most authors suggest that gender-based social-cultural factors lead to higher rates of suicidal behaviour among women in LMICs and, thus, to relatively high female suicide rates. We aim to test an alternative hypothesis: differences in the method and case-fatality of suicidal behaviour – *not* differences in the rates of suicidal behaviour – are the main determinants of higher female suicide rates in LMICs.

**Methods:**

A prospective registry of suicide attempts treated in all 14 general hospitals in a rural county in China was established and data from the registry were integrated with population and mortality data from the same county from 2009 to 2014.

**Results:**

There were 160 suicides and 1010 medically-treated suicidal attempts in the county; 84% of female suicides and 58% of male suicides ingested pesticides while 73% of female attempted suicides and 72% of male attempted suicides ingested pesticides. The suicide rate (per 100 000 person-years of exposure) was 8.4 in females and 9.1 in males (M:F ratio = 1.08:1) while the incidence of ‘serious suicidal acts’ (i.e. those that result in death or received treatment in a hospital) was 81.5 in females and 47.7 in males (M:F ratio = 0.59:1). The case-fatality of serious suicidal acts was higher in males than in females (19 *v.* 10%), increased with age, was highest for violent methods (92%), intermediate for pesticide ingestion (13%) and lowest for other methods (5%).

**Conclusions:**

The incidence of medically serious suicidal behaviour among females in rural China was similar to that reported in HICs, but the case-fatality was much higher, primarily because most suicidal acts involved the ingestion of pesticides, which had a higher case-fatality than methods commonly used by women in HICs. These findings do not support sociological explanations for the relatively high female suicide rate in China but, rather, suggest that gender-specific method choice and the case-fatality of different methods are more important determinants of the demographic profile of suicide rates. Further research that involves ongoing monitoring of the changing incidence, demographic profile and case-fatality of different suicidal methods in urban and rural parts of both LMICs and HICs is needed to confirm this hypothesis.

## Introduction

Suicide is a major public health problem worldwide, but suicide rates and the male-to-female ratio of suicide rates vary greatly between countries (WHO, 2014). Unlike most high-income countries (HICs) where the male-to-female ratio of suicide rates is 3:1 or higher, the reported gender ratio in China ranges from 0.9:1 to 1.4:1 (WHO, 2014; Jiang *et al*., 2018). Thus to achieve the Sustainable Development Goal (SDG) of decreasing suicide rates by 33% from 2015 to 2030 (UN, 2015), China must identify the causes of the relatively high suicide rate in females and take appropriate preventative action. This issue also needs to be addressed in other low- and middle-income countries (LMICs) with high rates of female suicide, such as India (India State-Level Disease Burden Initiative Suicide Collaborators, 2018).

Several researchers argue that population structure imbalance due to selective abortion of females (Yip and Liu, 2006) or high female labour force participation rates (Chen *et al*., 2017) contributes to the high female suicide rate in China. Other authors focus on the role of poverty (Lemmi *et al*., 2016) and socioeconomic inequity (Lorant *et al*., 2018). Such socio-economic explanations assume that gender-specific stressors in China lead to more frequent suicidal behaviour in females, and, thus, higher female suicide rates. There is, however, no evidence supporting the assumption that suicidal behaviour is more common in Chinese females than among females in HICs. Suicide rates are determined both by the incidence of different methods of suicidal acts and by the case-fatality of the different methods, so national differences in female suicide rates do not necessarily imply different rates of female suicidal behaviour, they could also be due to the use of different methods that have different case-fatality.

In almost all countries, the rates of non-fatal suicidal behaviour are much higher in females than in males, while the rates of death by suicide are higher in males than females (Hawton and Harriss, 2008; Perry *et al*., 2012; Mergl *et al*., 2015; Han *et al*., 2016). This indicates that the case-fatality of suicidal behaviour is greater in men than in women, presumably because men tend to choose methods that have a higher case-fatality. This assumption has been confirmed in the few HICs that have population-based registries of suicidal behaviour which make it possible to estimate method-specific case-fatality (Perry *et al*., 2012; Mergl *et al*., 2015). Several researchers have shown that the inverse male-to-female ratios between non-fatal and fatal suicidal behaviour are directly related to the much higher case-fatality of suicidal behaviour in males (Elnour and Harrison, 2008; Hawton and Harriss, 2008).

Identifying the causes for the low male-to-female suicide ratio in many LMICs and developing targeted interventions to address the relatively high rates of female suicide in these countries require establishing ongoing population-based registries of both fatal and non-fatal suicidal acts that can be used to estimate the gender-specific incidence and case-fatality of the most common methods of suicidal behaviour. To our knowledge, no such registry has been previously reported in China. The current paper describes a hospital-based registry of suicidal acts that operated from 2009 to 2014 in one county in Shaanxi Province. Combining this registry data with population data and suicide mortality data from the county made it possible to estimate the gender-specific incidence and case-fatality of different types of ‘medically serious suicidal behaviour’ (i.e. suicidal acts that result in death or require treatment in a hospital).

## Methods

### Study setting

This study was conducted in Meixian County of Shaanxi Province, a province in the central western part of the country with a per capita GDP which ranks in the middle of 31 provinces in mainland China. Meixian is a rural county consisting of ten townships with a population of about 300 000, 80% of whom earn their livelihood by farming. Meixian County is one of the national Disease Surveillance Points under the national Centers for Disease Control (CDC) which uses standard procedures for monitoring all deaths. The suicide rate in the county and the proportions of suicides due to pesticide ingestion are similar to those reported in other parts of rural China. There are two county-level general hospitals and 12 township-level general hospitals; these 14 hospitals are the only medical centres that provide resuscitation services for medically serious injuries, including all medically serious suicide attempts.

### Data sources

All self-harm injuries of persons 10 years of age or older treated in the 14 general hospitals from 1 January 2009 through 31 December 2014 were prospectively recorded in the self-harm registry. Data from the death reporting system maintained by the Meixian County CDC (one of China's 161 ‘Disease Surveillance Points’ that has standardised procedures for registering deaths (Sha *et al*., 2018)) from 2009 through 2014 for deaths assigned ICD-10 codes of X60–X84, Y10–Y34, Y87 (i.e. death by suicide) were identified. Population data from the Meixian County Bureau of Statistics were used to estimate the person-years of exposure between 2009 and 2014.

### Measures

Information about the gender and age of the target individual and the date and method of the index act of self-harm was obtained by trained researchers on all cases of self-harm treated at the 14 hospitals and all deaths recorded as suicides in the county-level mortality dataset. Each act of self-harm was initially classified as suicide, suicide attempt or non-suicidal self-harm (i.e. self-harm without intention to die, as assessed by the researcher who interviewed the individual and other informants). After excluding the cases of non-suicidal self-harm, multiple records of the same suicidal act (e.g. when seen in multiple hospitals or when appearing both in hospital records and in the death registry) were merged into a single record and classified as ‘suicide attempt’ if the individual survived or ‘suicide’ if the individual died. Suicidal acts reported in the hospital registry that resulted in death within 1 week without a second intervening suicidal act were classified as a suicide.

The person-years of exposure to the risk of suicide and suicide attempt for the total population and for the different population subgroups assessed (stratified by gender and age group) were estimated as the sum of the annual midpoint population over the 6 years of follow-up.

### Statistical analysis

Separate records were made for each suicidal act in individuals who made multiple suicidal acts over the 6-year follow-up. We divided suicidal methods into five groups: pesticide ingestion, ingestion of medications, cutting and stabbing injuries, other violent methods (including hanging, jumping, drowning or burning) and other methods (e.g. other poisons).

We estimated the mean annual rates of suicide and the mean annual incidence of medically treated suicide attempts using the total person-years of exposure over the 6 years. Stratified estimates by method, gender and age group (10–34, 35–59, 60 or older) were made using the person-years of exposure in each cohort. Case-fatality ratios for ‘medically serious suicidal behaviour’ (defined as suicidal acts that either resulted in death or received hospital treatment) for different population cohorts and different methods of suicide were computed as the proportion of all suicidal acts in the cohort that resulted in death (i.e. suicides/(suicides + attempted suicides)). The Poisson distribution was used to estimate 95% confidence intervals (95% CIs) of the estimates, a *χ*^2^ for linear trend was used to test whether there was a stepwise change in case-fatality with age, and a Tukey-type multiple comparison test was used to compare the proportional distribution of the different methods of suicide by gender (Zar, 1999).

## Results

There were 1 827 839 person-years of potential risk for suicidal behaviour in Meixian from 2009 to 2014. As shown in Fig. 1, 160 suicides and 1010 medically treated, non-fatal suicide attempts occurred in the country over this 6-year period. Among 1110 suicidal acts which received medical treatment, 9.0% (100/1110) were not successfully resuscitated; resuscitation failed in 75.0% (9/12) of suicidal acts by violent methods (hanging, jumping, drowning and burning), 10.3% (84/817) by pesticide ingestion, 2.4% (4/165) by ingesting medications, 1.7% (1/59) by cutting injuries; and 3.5% (2/57) by other methods. Among the 998 individuals who made a medically treated, non-fatal suicide attempt, 12 (1.2%) made a second non-fatal attempt and 23 (2.3%) died following a subsequent suicidal act during the 6-year period.

**Fig. 1.** Identification of suicides and medically treated, non-fatal attempted suicides in Meixian County, Shaanxi Province, China: 2009–2014.

The gender, age and method of suicides and medically treated suicide attempts are shown in Table 1. Compared to the 975 individuals who attempted suicide and did not subsequently die by suicide during the follow-up period, individuals who died by suicide were older (mean [s.d.] age 48.0 [18.0] *v.* 38.6 [16.5], *t* = 6.16, *p* < 0.001) and more likely to be male. In both groups, the dominant method was ingestion of pesticides – accounting for over 70% of all suicide deaths and suicide attempts. Among the less common methods, suicide decedents were more likely to use a violent method (i.e. hanging, jumping, drowning or burning), while suicide attempters were more likely to use less violent methods (i.e. ingestion of medications or cutting).

**Table 1.** Demographic characteristics of suicide decedents and suicide attempters in Meixian County, Shaanxi, China: 2009–2014

Characteristic	Age, gender and method of all medically treated suicide attempts		Age, gender and method of the first attempt in medically treated attempters who did not subsequently die of suicide^a^		Age, gender and method of suicide decedents		Comparison of age, gender and method of suicide decedents to those of the first attempt in medically treated suicide attempters who did not subsequently die of suicide	
	(*N* = 1010)		(*N* = 975)		(*N* = 160)			
	*n*	%	*n*	%	*n*	%	*χ*^2^	*p*
**Age group**							32.46	<0.001
10–34	456	45.1	444	45.5	46	28.8		
35–59	413	40.9	399	40.9	66	41.3		
⩾60	141	14.0	132	13.5	48	30.0		
**Gender**							18.29	<0.001
Female	644	63.8	624	64.0	74	46.3		
Male	366	36.2	351	36.0	86	53.8		
**Method**							204.14	<0.001
Pesticide	733	72.6	708	72.6	112	70.0		
Medication	161	15.9	154	15.8	7	4.4		
Cutting or stabbing	58	5.7	57	5.8	3	1.9		
Other violent methods^b^	3	0.3	3	0.3	34	21.3		
Other methods^c^	55	5.4	53	5.4	4	2.5		

a This group of unduplicated individuals with suicide attempts does not overlap with the suicide decedent group and, thus, can be compared with the suicide decedents using standard statistical tests.

b Includes hanging, jumping, drowning and burning.

c Includes other types of poisons and miscellaneous methods.

As shown in Table 2, the mean suicide rate over the 2009–2014 time period was 8.8 per 100 000 person-years, the incidence of medically treated suicide attempts was 55.3, and the incidence of all medically serious suicidal acts was 64.0. The suicide rate was only slightly higher in males than in females (M:F ratio of suicide rates = 1.08:1) but the incidence of suicide attempts was much higher in females than in males (M:F ratio = 0.53:1), resulting in a significantly higher case-fatality for suicidal acts among males than females (19.0 *v.* 10.3%; *χ*^2^ = 17.87, *p* < 0.001). The suicide rate shows a strong stepwise increase by age while the incidence of suicide attempts is highest in the youngest age group (10–34 years of age) and lowest in the middle age group (35–59 years of age). The case-fatality of suicidal acts shows a significant stepwise increase with age (*χ*^2^for trend = 27.98, *p* < 0.001).

**Table 2.** Suicide rates, incidences of medically treated suicide attempts and suicidal acts, and the case-fatality of suicidal acts among different population cohorts in Meixian County, Shaanxi, China: 2009–2014

Population	Cumulative person-years^a^	Suicide deaths *n*	Suicide rate per 100 000 person-years (95% CI)	Medically treated suicide attempts *n*	Incidence of suicide attempt per 100 000 person-years (95% CI)	Suicidal acts (suicide deaths plus attempts) *n*	Incidence of suicidal acts per 100 000 person-years (95% CI)	Case-fatality of suicidal acts % (95% CI)
Total	1 827 839	160	8.8 (7.5–10.2)	1010	55.3 (51.9–58.8)	1170	64.0 (60.4–67.8)	13.7 (11.7–15.6)
**Gender**								
Female	881 114	74	8.4 (6.6–10.5)	644	73.1 (67.6–79.0)	718	81.5 (75.6–87.7)	10.3 (8.1–12.5)
Male	946 725	86	9.1 (7.3–11.2)	366	38.7 (34.8–42.8)	452	47.7 (43.5–52.4)	19.0 (15.4–22.6)
**Age group**								
10–34	672 354	46	6.8 (5.0–9.2)	456	67.8 (61.7–74.3)	502	74.7 (68.3–81.5)	9.2 (6.6–11.7)
35–59	727 233	66	9.1 (7.0–11.6)	413	56.8 (51.4–62.5)	479	65.9 (60.1–72.0)	13.8 (10.7–16.9)
⩾60	230 171	48	20.9 (15.4–27.7)	141	61.3 (51.6–71.3)	189	82.1 (70.8–94.7)	25.4 (19.2–31.6)

a Cumulative person-years of exposure is the estimated mid-year population summed over the 6 years of follow-up (2009 through 2014).

Table 3 shows that the methods used in suicide attempts were similar by gender (*χ*^2^ = 7.43, df = 4, *p* = 0.115): for both males and females more than 70% of attempts involve the ingestion of pesticides, the second most common method is the ingestion of medications, violent methods were quite uncommon, and the other methods (i.e. cutting and miscellaneous methods) accounted for <15% of all cases. However, the methods used in fatal suicidal acts varied significantly by gender (*χ*^2^ = 14.14, df = 4, *p* = 0.007): females were more likely to die by pesticide ingestion while males were more likely to die by violent methods (Tukey-type multiple comparison, *q*(5 groups) = 4.70, *p* < 0.01).

**Table 3.** Proportions of different methods used in suicides and suicide attempts, and the incidence and the case-fatality of different methods of suicide

Suicidal method	Medically treated suicide attempt				Suicide				Incidence of suicidal acts per 100 000 person-years			Case-fatality^a^		
	Female		Male		Female		Male		Female (95% CI)	Male (95% CI)	Total (95% CI)	Female	Male	Total
	*n*	%	*n*	%	*n*	%	*n*	%				% (95% CI)	% (95% CI)	% (95% CI)
Pesticide	469	72.8	264	72.1	62	83.8	50	58.1	60.3 (55.3–65.56)	33.2 (29.6–37.1)	46.2 (43.2–49.4)	11.7 (8.9–14.4)	15.9 (11.9–20.0)	13.3 (11.0–15.5)
Medication	107	16.6	54	14.8	3	4.1	4	4.7	12.5 (10.3–15.1)	6.1 (4.7–7.9)	9.2 (7.9–10.7)	2.7 (0.5–6.6)	6.9 (1.8–14.8)	4.2 (1.7–7.7)
Cutting or stabbing	38	5.9	20	5.5	0	0.0	3	3.5	4.3 (3.1–5.9)	2.4 (1.5–3.7)	3.3 (2.6–4.3)	0.0 (0.0–2.5)	13.0 (2.7–29.5)	4.9 (1**.**0–11.7)
Other violent methods^b^	3	0.5	0	0.0	8	10.8	26	30.2	1.3 (0.6–2.2)	2.8 (1.8–4.0)	2.0 (1.4–2.8)	72.7 (44.1–93.7)	100.0 (96.4–100.0)	91.9 (81.1–98.4)
Other methods^c^	27	4.2	28	7.7	1	1.4	3	3.5	3.2 (2.1–4.6)	3.3 (2.2–4.7)	3.2 (2.5–4.2)	3.6 (0.0–13.4%)	9.7 (2.0–22.3)	6.8 (1.8–14.5)

a Case-fatality was calculated as the numbers of suicide deaths divided by the numbers of suicidal acts (i.e. suicide deaths plus suicide attempts).

b Includes hanging, jumping, drowning and burning.

c Includes other types of poisons and miscellaneous methods.

Combining suicides and suicide attempts to assess ‘medically serious suicidal acts’, the incidence of suicidal acts using violent methods was significantly higher in men than in women (2.7 *v.* 1.2 per 100 000 person-years, *Z* = 2.28, *p* = 0.023), but the incidence of serious suicidal acts by pesticide ingestion, medication ingestion, and cutting or stabbing were significantly higher in women than in men (60.3 *v.* 33.2, *Z* = 8.43, *p* < 0.001; 12.5 *v*. 6.1, *Z* = 4.43, *p* < 0.001; and 4.3 *v.* 2.4, *Z* = 2.18, *p* = 0.029, respectively).

The case-fatality of violent suicidal methods was 92% (34/37), the case-fatality of pesticide ingestion was 13% (112/845), and the case-fatality of the other three classes of methods considered ranged from 4 to 7% and averaged 5% (14/288). For all five methods of suicide, case-fatality was higher in males than in females, but this difference was only statistically significant for violent methods (Fisher exact test *p* = 0.021) and for cutting and stabbing (Fisher exact test *p* = 0.049), not for pesticide ingestion (15.9 *v.* 11.7%, *χ*^2^ = 3.10, *p* = 0.078).

## Discussion

### Main findings

This study integrated 6 years of prospectively collected population data, suicide mortality data and hospital registry data from one rural county in China. Based on the 1.8 million person-years of exposure, we identified several key findings not previously reported in China: (a) the male-to-female ratio of the incidence of ‘medically serious suicidal acts’ (i.e. those resulting in death or treatment in a hospital) (0.59:1) was similar to that reported in other countries, but the male-to-female ratio of suicide death rates (1.08:1) was much lower than reported elsewhere; (b) the incidence of suicidal acts by pesticide ingestion was higher in women than in men, but the incidence of violent suicidal acts (i.e. hanging, jumping, drowning or burning) was higher in men than in women; (c) the overall case-fatality of medically serious suicidal acts was significantly higher in men than in women (19 *v.* 10%); (d) the method-specific case-fatality for all five groups of suicidal methods was also higher in men, but the difference was not statistically significant for pesticide ingestion; and (e) medical resuscitation of suicidal acts involving pesticide ingestion fails in 10% of cases. Other findings confirmed reports from previous studies: suicide decedents were older than individuals with medically treated, non-fatal suicide attempts; the proportion of females among those who attempted suicide was much higher than the proportion of females among those who died by suicide; the case-fatality of suicidal acts increased with age; and pesticide ingestion was the dominant form of medically serious suicidal behaviour in this rural agricultural community, accounting for 70% of all suicides and 73% of all medically treated suicide attempts.

### Strengths and limitations

Village doctors in Meixian County who encounter acute self-harm injuries always send them directly to the local hospital, emergency department staff of all 14 hospitals in the county were trained to register all cases of self-harm, emergency services for all county residents were provided at these 14 hospitals, and research staff made regular visits to participating hospitals to monitor case collection; so virtually all acts of self-harm in the county that resulted in medical treatment over the 6-year follow-up period were identified. Cases were carefully reviewed to exclude the cases of non-suicidal self-injury, to combine multiple reports of the same suicidal act and to definitively classify each suicidal act either as a suicide or as a non-fatal suicide attempt. We did not, however, independently assess the completeness of suicidal deaths reported in the county's death registry system, but Meixian County is one of the national ‘Disease Surveillance Points’ managed by the national CDC which monitors its death registry system. These procedures made it possible to provide estimates that have previously not been available in China: the incidence of medically treated suicide attempts, the incidence of medically serious suicidal acts (i.e. those that result in death or receive treatment in a hospital) and the case-fatality of medically serious suicidal acts both for the entire population and stratified by gender, age and method of suicide.

Several caveats should be considered when assessing these results. The suicide rate and proportion of suicides by pesticide ingestion in Meixian County are similar to the estimates of suicide rates and of the proportion of suicides by pesticide ingestion for all of rural China (Page *et al*., 2017; Jiang *et al*., 2018), but we cannot be certain how representative Meixian is of all rural China. Less serious suicidal acts in the community do not receive medical treatment (Geulayov *et al*., 2018), so the results are only relevant to persons who die of suicide or receive medical treatment for suicidal acts. Despite being part of the national Disease Surveillance Points system, the failure to report 27 of the suicides we identified at hospitals in Meixian's CDC death registry system suggest that under-reporting (and, possibly, misclassification) of suicides is a problem (this happens in almost all jurisdictions); under-reporting of suicide deaths by the CDC would mean that our reported case-fatality ratios are somewhat lower than the actual case-fatality ratios. All reported results are combined over the 6-year period so we were unable to monitor trends in the rates over time. Finally, the specific pesticide(s) employed in the suicidal act was only identified in a minority of cases, so it was not possible to compare the case-fatality of different types of pesticides.

### Pesticide ingestion and China's low male-to-female ratio of suicide rates

The relatively high suicide rate among rural Chinese women and the corresponding low male-to-female ratio of suicide rates in rural China are *not* due to high rates of suicidal behaviour among rural women. The incidence of suicidal acts in rural women (81.5 per 100 000 person-years) is similar to or lower than that reported elsewhere (Perry *et al*., 2012; Mergl *et al*., 2015; Han *et al*., 2016), so the long list of sociocultural factors previously considered explanations for the high rate of suicide in rural Chinese females (Lemmi *et al*., 2016; Lorant *et al*., 2018) are unlikely to be the most important determinants. We conclude that the most important determinant is the high 10% case-fatality of medically serious suicidal acts in rural Chinese women, which is twofold to tenfold higher than the 1–5% female case-fatality of suicidal acts reported in HICs (Elnour and Harrison, 2008; Hawton and Harriss, 2008; Mergl *et al*., 2015; Han *et al*., 2016). This high case-fatality in rural Chinese women is, in turn, driven by the large proportion of suicidal acts involving the ingestion of pesticides, which has a case-fatality in females of 12%.

As is true in most locations (Elnour and Harrison, 2008; Miller *et al*., 2012; Mergl *et al*., 2015; Han *et al*., 2016), rural Chinese men are much more likely than rural Chinese women to use violent suicidal methods that are highly lethal (with a 92% case-fatality). However, only 3% (37/1170) of medically serious suicidal acts use these violent methods in rural China, so the influence of suicides involving violent methods on the gender ratio is limited. On the other hand, despite a somewhat lower case-fatality for suicidal acts involving pesticide ingestion among women than men (12 *v.* 16%), the much larger number of women who use this method (531 women *v.* 314 men in this sample) results in a greater number of fatal pesticide ingestion suicides among women than among men (62 *v.* 50). This increases the female suicide rate and largely negates the effect of the higher number of violent suicide deaths in men than women (26 *v.* 8); the relatively higher female suicide rates result in decreasing the male-to-female ratio of suicide rates towards a 1:1 ratio. The Chinese population is now about 43% rural (National Bureau of Statistics of China, 2017) and rural suicide rates are approximately twice that of urban rates (Jiang *et al*., 2018), so the demographic characteristics of rural suicides have a substantial effect on China's national suicide rate, resulting in a much higher female suicide rate and a much lower male-to-female ratio of suicide rates for China as a whole than for most other countries (WHO, 2014).

In urban areas of China, suicides and suicide attempts involving pesticide are uncommon, presumably because these agents are not readily available. In these settings, the method of choice of suicidal acts is closer to that reported in Western countries, with hanging, jumping and ingestion of medication replacing the pesticide ingestion cases seen in rural areas (Xu *et al*., 2013; Page *et al*., 2017). There are currently no population-based studies from urban areas of China comparable to the current study from rural China that could provide case-fatality estimates of suicidal acts by method and by gender, but we expect that in the absence of pesticides, a higher proportion of urban men than rural men employ violent suicidal methods with high case-fatality ratios, while a higher proportion of urban women than rural women employ suicidal methods with low case-fatality ratios such as medication ingestion and cutting or stabbing. Assuming no substantial change in the male-to-female ratio of the incidence of medically serious suicidal acts over time, these gender-based changes in the preferred method of suicide during urbanisation would result in a relatively faster decrease in female suicide rates and a corresponding gradual increase in the male-to-female ratio of suicide deaths. Jiang *et al.* (2018) reported that from 2002 to 2015, the national male-to-female ratio of suicide deaths increased from 1.1 to 1.4. This transformation in the gender ratio of suicide has occurred over the last 25 years in China as the population has changed from 20% urban in 1990 to 57% urban in 2016 (National Bureau of Statistics of China, 2017).

We predict that as China continues to urbanise and as an increasing proportion of the rural population is no longer engaged in agricultural production the national female suicide rate will continue to decline and the male-to-female ratio of suicide rates will continue to increase. We also predict that in other LMICs where pesticide ingestion is a common method of suicide in rural communities, ongoing urbanisation will be associated with relatively faster decreases in female suicide rates and corresponding increases in the male-to-female ratio of suicide rates.

### Implications for suicide prevention in China and other LMICs

Despite a substantial decrease in the estimated proportion of global suicides due to pesticide ingestion over the last decade (Gunnell *et al*., 2007; Mew *et al*., 2017), pesticide ingestion remains the dominant method of suicide and attempted suicide in rural China and a common method of suicide in rural parts of many other LMICs (Gunnell *et al*., 2007; Mew *et al*., 2017; Page *et al*., 2017). Reducing pesticide ingestion suicides in these countries is an important part of the national suicide prevention effort that will require: (1) ongoing monitoring of the incidence, case-fatality and demographic profile of different types of suicidal behaviour; (2) bans on the production of the most hazardous pesticides (WHO, 2019); (3) reducing access to the most lethal pesticides; (4) improving the medical treatment of pesticide ingestion in rural health centres; and (5) promoting safety consciousness among rural residents. Given substantial differences in the lethality of different pesticides, registry systems of fatal and non-fatal suicidal behaviour must include information on the specific types of pesticides employed in suicidal acts.

Several researchers and experts have suggested that providing household- or community-based lockboxes for pesticides to restrict access should reduce suicide rates (Konradsen *et al*., 2007; WHO, 2016), but the definitive study on this mean restriction method of preventing suicides in Sri Lanka did *not* find any reduction in suicide rates (Pearson *et al*., 2017). We believe that the effort to restrict access should now shift to top-down approaches (including the restriction of production of the most potent pesticides, development of less toxic pesticides, scaled taxation of pesticides based on the lethality of the product, package size limitations, training pesticide vendors, etc. (Eddleston *et al*., 2012; Gunnell *et al*., 2017; Weerasinghe *et al*., 2018)) rather than depending on bottom-up approaches such as pesticide lockboxes that require the ongoing active participation of community members. The relatively high proportion of suicidal acts involving pesticide ingestion that result in death despite receiving treatment in a local hospital (10.3%), a finding that was similar with a previous study in Sri Lanka (Eddleston *et al*., 2006), indicates the importance of improving the training of medical staff and the access to necessary medical equipment in rural community health centres where pesticide ingestion suicides are commonly treated (WHO, 2008).

Consistent with previous studies (Elnour and Harrison, 2008; Hawton and Harriss, 2008; Han *et al*., 2016), the case-fatality of suicidal acts in our study increased with the age – over one in four medically serious suicidal acts in individuals over 60 years of age were fatal while less than one in ten in individuals under 35 were fatal. This highlights the need to put proportionally more resources on suicide prevention among the elderly.

Major changes in the methods used in suicidal acts that occur with rapid urbanisation have a substantial effect on the rate and demographic pattern of suicide that offer potential opportunities for suicide prevention. But very few LMICs collect population-based data on the method-specific incidence of both fatal and non-fatal suicidal behaviour that could be used to take advantage of this opportunity. The World Health Organization Global Suicide Report strongly recommends that countries and sub-national localities establish hospital-based registries of medically treated suicide attempts that can be integrated with suicide mortality data to assess trends in the demographic distribution and case-fatality of different methods over time (WHO, 2014). We consider this an essential component of national and local suicide prevention efforts in China and in other LMICs. Polices informed by the information provided by such registries that effectively limit access to pesticides – which remain an important factor in rural suicides in China and many other LMICs – are needed.

## Data

This is one report on a dataset for which additional publications are still in preparation. When all the main papers from the dataset have been published, the original dataset will be provided to interested readers on request.
